# Serum Magnesium in Patients With Acute Myocardial Infarction and Its Effect on Cardiac Complications and Mortality in Myocardial Infarction Patients

**DOI:** 10.7759/cureus.38147

**Published:** 2023-04-26

**Authors:** Zia Sabah, Javed Wani, Mosab Deajim, Ahmed S AL Zomia, Abdullah Asiri, Ali A Alqahtani, Wasna Alansari, Amin Alwan, Ryan M AL Qahtani, Berin Raj

**Affiliations:** 1 Medicine, King Khalid University, Abha, SAU; 2 Internal Medicine, King Khalid University, Abha, SAU; 3 Medicine and Surgery, King Khalid University, Abha, SAU; 4 Medicine, King Saud Bin Abdulaziz University for Health Sciences, Jeddah, SAU; 5 Family and Community Medicine, King Fahad General Hospital, Gizan, SAU; 6 Epidemiology and Public Health, Prince Faisal Bin Khalid Cardiac Center, Abha, SAU

**Keywords:** cardiac complications, mortality, outcomes, mi, serum magnesium

## Abstract

Background

Magnesium is an essential micronutrient for people and is crucial in maintaining healthy cardiac function. It functions as a cofactor in a number of the body's enzyme systems, and myocardial cells are one of its target tissues. The upkeep of the myocardium's normal functional integrity depends on a lot of things including magnesium ions.

Magnesium plays an important role in the pathophysiology of cardiovascular disorders.

Aim

This study aims to estimate serum magnesium levels and their correlation with cardiac complications and mortality in patients with acute myocardial infarction (AMI).

Methods

Patients with acute myocardial infarction who visited the Prince Faisal Bin Khalid Cardiac Center within 12 hours of the onset of symptoms were the subjects of this study. On the first and fifth days following admission, the level of serum magnesium was assessed. Statistical Package for Social Sciences (SPSS) version 20 (IBM SPSS Statistics, Armonk, NY) was used to analyze the collected data.

Results

The current study comprised 160 patients with acute myocardial infarction; there were 84 (52.5%) who experienced a low level of serum magnesium on admission. Significantly higher proportions of patients who experienced low magnesium levels had diabetes mellitus (P=0.0072) and a history of diuretics (P=0.03) and were administrated beta-blockers (P=0.01), calcium channel blockers (P=0.04), and statins (P=0.007) after admission. Significantly higher proportions of patients with low serum magnesium experienced atrial fibrillation (P=0.03), angina (P=0.03), and cardiogenic shock (P=0.003).

Conclusion

Low magnesium levels are associated with poor outcomes in most patients admitted with acute myocardial infarction.

## Introduction

Magnesium is an essential element of the functioning human body; it is naturally present in many foods and is also available as a dietary supplement. An adult's body contains almost 24 g of magnesium, with 50%-60% present in the bones and the rest present in soft tissues. The serum magnesium level represents less than 1% of the total body magnesium [1].

Magnesium serves as a cofactor for more than 300 enzymatic reactions, such as those responsible for glycemic control, blood pressure, and lipid peroxidation [2]. Its possible site of action involves platelets, smooth muscles, and myocardial cells. The deficiency of magnesium can evoke hyperlipidemia and, subsequently, atherogenic deposits in coronary arteries leading to atherosclerosis [2]. Hence, it is crucial for the cardiovascular system [1].

Magnesium is also essential for human beings as it plays an important role in myocardial physiology [3]; low magnesium concentration within the myocardial cell is associated with membrane destabilization, whereas high concentrations are membrane stabilizing and, therefore, antiarrhythmic [3]. Minor changes in the physiologic concentrations of ions can have catastrophic outcomes [4]. Magnesium has been stated to have an effect on the occurrence of acute myocardial infarction (AMI) and its sequelae, such as arrhythmia. Also, it has a great role in the pathogenesis of other cardiovascular diseases [5].

AMI is a major health issue in industrial countries and is becoming an increasingly important problem in developing countries [6]. In myocardial infarction (MI), a functional deficit of available magnesium occurs due to the trapping of free magnesium in adipocytes [7]. It was indicated that the serum magnesium level is low in the first 48 hours following AMI and later rises gradually to attain the normal level in almost three weeks [5]. Therefore, this study was conducted to evaluate the serum magnesium levels and their correlation with cardiac complications and mortality in patients with acute myocardial infarction who presented within 12 hours of the onset of symptoms.

## Materials and methods

Subjects and ethics

This study was conducted in the year 2022 over a period of six months on patients with acute myocardial infarction who presented at the hospital within 12 hours of the onset of symptoms. The diagnosis of acute myocardial infarction was based on the presence of two of the three following criteria: history of discomfort in the chest, changes in the ECG suggestive of acute myocardial infarction, and rise of cardiac enzymes. On the other hand, patients who had hypokalemia and patients who did not fulfill the previous criteria for acute myocardial infarction diagnosis were excluded. All the participating patients provided written consent before being involved in the study after an explanation of the probable benefits in the local language.

After receiving approval from the Research Ethics Committee of Prince Faisal Bin Khalid Cardiac Center and King Khalid University in Abha, Saudi Arabia, the study was carried out.

Examination and clinical analysis

As part of the assessment routine for any patient admitted with acute myocardial infarction in the ICU, patients had appropriate history and physical examinations and were undergoing biochemical analysis at the department of biochemistry at the cardiac center. All patients had full blood counts, urine tests, blood sugar, blood urea, serum creatinine, fasting lipid profiles, cardiac enzymes, and ECGs as part of the biochemical studies. On days 1 and 5 after admission, the serum magnesium level was estimated.

The serum magnesium level was estimated based on the fact that magnesium reacts with xylidyl blue at alkaline pH resulting in the formation of a chelating red-colored compound. The increase in the red color or the decrease in the blue color is proportionate to the concentration of magnesium in the serum. The estimation of magnesium was based on the colorimetric endpoint test with xylidyl blue as the reagent. The specimen used for magnesium was non-hemolyzed serum. The separation of serum from the cell was done as early as possible, and hemolysis was avoided. The normal range for serum magnesium is 1.6-2.4 mg/dL.

Statistical analysis

The collected data was entered into a Microsoft Excel spreadsheet (Microsoft® Corp., Redmond, WA), compiled, and exported to Statistical Package for Social Sciences (SPSS) version 20.0's data editor (IBM SPSS Statistics, Armonk, NY). Categorical variables were given as frequency and percentage, whereas continuous variables were expressed as mean±SD. Depending on the type of data, the chi-square test or Fisher's exact test was performed to ascertain the relationship between various variables. P-values lower than 0.05 were regarded as statistically significant.

## Results

A total of 160 patients were included in the current study; there were 84 (52.5%) who experienced a low level of serum magnesium on admission, whereas 76 (47.5%) experienced a normal level. The comparison between the two groups is shown in Table 1. The level of serum magnesium significantly varied between diabetic patients and those on diuretics; magnesium levels significantly tended to be low among diabetic patients (P=0.0072) and those on diuretics (P=0.03).

**Table 1:** Characteristics of included study population at the time of admission. Values are mean±standard deviation or percentages. HT, hypertension; DM, diabetes mellitus; MI, myocardial infarction; LAD, left anterior descending artery; LCX, left circumflex artery; LMCA, left main coronary artery; RCA, right coronary artery; Hb, hemoglobin; CK, creatine kinase; IU, international units; ACEIs, angiotensin-converting enzyme inhibitors; ARBs, angiotensin receptor blockers

Variable	Serum Magnesium Levels on Admission (mg/dL)		P-value
	<1.80 (n=84)	>1.80 and <2.60 (n=76)	
Age, Years	64.4±14.4	63.6±12.6	0.710
Sex, n (%)			
Male	65 (77)	62 (81)	0.537
Female	19 (23)	14 (19)	0.537
Comorbidities, n (%)			
HT	45 (53)	32 (42)	0.166
DM	43 (51)	23 (30)	0.007
Dyslipidemia	41 (49)	26 (34)	0.056
History of MI	20 (24)	26 (34)	0.164
Infarct-Related Vessel, n (%)			
LAD	43 (51)	40 (53)	0.801
LCX	12 (14)	9 (12)	0.709
LMCA	8 (10)	11 (14)	0.437
RCA	11 (13)	16 (21)	0.178
Laboratory Test Reports			
Hb, g/dL	12.6±3.4	13.2±2.3	0.198
Sodium, mEq/L	141.18±3.4	141.24±3.45	0.318
CK, IU/L	116.5±32	111.4±32.3	0.318
Ejection Fraction	42.9±16.2	41.3±15.6	0.526
History of Medication, n (%)			
Beta-blockers	9 (11)	6 (8)	0.521
ACEIs or ARBs	23 (27)	24 (32)	0.489
Aspirin	8 (10)	10 (13)	0.553
Clopidogrel	5 (6)	7 (9)	0.471
Statins	7 (8)	9 (12)	0.399
Diuretics	28 (33)	14 (18)	0.031

The correlation between the level of magnesium and medication post-admission was investigated (Table 2). Higher proportions of patients administrated with beta-blockers (71%), calcium channel blockers (32%), and statins (88%) significantly tended to display a low level of serum magnesium: P=0.019, 0.04, and 0.007, respectively.

**Table 2:** Medication post-admission. Values are expressed in numbers (%). ACEIs, angiotensin-converting enzyme inhibitors; ARBs, angiotensin receptor blockers

Medicine	Serum Magnesium Levels on Admission (mg/dL)		P-value
	<1.80 (n=84)	>1.80 and <2.60 (n=76)	
Aspirin	73 (87)	63 (83)	0.479
Clopidogrel	41 (49)	35 (46)	0.705
Βeta-blockers	60 (71)	40 (53)	0.019
ACEIs or ARBs	46 (55)	35 (46)	0.257
Calcium Channel Blockers	27 (32)	14 (18)	0.043
Statins	74 (88)	54 (71)	0.008
Ticagrelor	30 (36)	24 (32)	0.595

The assessment of the correlation between the level of serum magnesium and in-hospital clinical outcomes (Table 3) showed that the level of serum magnesium significantly tended to be low among patients with atrial fibrillation (P=0.03), angina (P=0.03), and cardiogenic shock (P=0.003).

**Table 3:** In-hospital clinical outcome. Values are expressed in numbers (%). Sample size: 160 Significant level set: P<0.05 MI: myocardial infarction

Outcome	Serum Magnesium Levels on Admission (mg/dL)		P-value
	<1.80 (n=84)	>1.80 and <2.60 (n=76)	
Atrial Fibrillation	17 (20)	6 (8)	0.031
Angina (Post MI)	21 (25)	9 (12)	0.036
Ventricular Tachycardia	17 (20)	12 (16)	0.513
Ventricular Fibrillation	12 (14)	10 (13)	0.854
Thrombotic Events	5 (6)	3 (4)	0.565
Cardiogenic Shock	32 (38)	13 (17)	0.003
Sustained Premature Ventricular Beats	11 (13)	7 (9)	0.423

## Discussion

Magnesium deficiency is an issue for those who have coronary heart disease (CHD) [3]. Magnesium has also been reported to have an effect on AMI etiology [5]. As a result, the purpose of this study was to evaluate serum magnesium levels and how they are related to cardiac problems in AMI patients.

The normal level of magnesium was reported to be between 1.7 and 2.2 mEq/L; a serum level of less than 1.7 mEq/L is taken as a reference [3]. However, in the current study, we used mg/dL as the unit for measuring serum magnesium; therefore, the normal range for serum magnesium was set at 1.6-2.4 mg/dL. In our study, we found that more than one-half of patients (52.5%) showed a low level of serum magnesium on admission (<1.8 mg/dL).

In an Indian study, the comparison between the serum magnesium level between the control group and the acute myocardial infarction group showed that the mean level of serum magnesium among the group of patients was 1.01 with a range of 0.42-1.56, and it was considerably lower (P<0.01) compared to the control group (2.2 mEq/L) [3]. Although we did not compare our findings among AMI patients with the control group, the findings showed that AMI patients experienced a low level of serum magnesium, which was in agreement with the previous study [3].

A previous study revealed that serum magnesium was lower in AMI cases at admission within 24 hours compared to matched controls [6]. Another study conducted on AMI patients displayed that on the first day of admission, there were 16% and 34% of patients who experienced levels of serum magnesium of less than 1.6 and 1.6-2.4 mg/dL, respectively [5]. Our findings revealed that a higher proportion of patients (more than one-half) displayed low serum levels compared to the previous study [5].

According to a report, low magnesium may be caused by a number of things, including insufficient magnesium intake, ongoing stress, malabsorption, and medications such as diuretics [8]. This was in agreement with our findings as we found that a significantly higher proportion of AMI patients were administrating diuretics when assessing their history.

A study conducted on 465 consecutive AMI patients complicated with malignant ventricular arrhythmia categorized patients into two groups based on the serum magnesium level. More patients who reported a serum magnesium level of ≤2.3 mg/dL significantly experienced dyslipidemia, higher level of hemoglobin, and lower serum sodium and tended to administrate beta-blockers, angiotensin-converting enzyme inhibitors (ACEIs) or angiotensin receptor blockers (ARBs), calcium channel blockers, and statin after admission [9]. These findings showed agreement and contrast with our findings; in agreement with our findings, we found that a higher proportion of AMI patients were suffering from dyslipidemia; however, the significance level was not definite (P=0.05). On the other hand, the level of sodium was not varied significantly between the two groups regarding the level of serum magnesium, and although the mean level of hemoglobin was lower among AMI patients with low serum magnesium levels, there was no significant difference. Therefore, we did not find any association between the level of serum magnesium and hemoglobin and sodium level, and this was in contrast to the previous study [9].

Additionally, after admission, significantly higher proportions of AMI patients were treated with beta-blockers, calcium channel blockers, and statin, and this was in agreement with the previous study [9], but the disagreement was found regarding ACEI or ARB treatment after admission, as we found no significant difference between those with a low or normal level of serum magnesium level.

It was reported that individuals managed by intravenous magnesium post infarction were at a significantly lower risk of dying from ischemic heart disease-related complications [10,11]. However, there were no mortality cases reported in our study. Additionally, a study by Akila et al. conducted on AMI patients revealed that those patients with low magnesium levels were more predisposed to get arrhythmia [5]. Also, there were no arrhythmia cases reported in our study.

A study conducted on 9005 patients with AMI revealed that serum magnesium levels at 2.2 to ≤2.4 and more than 2.4 mg/dL were both significant predictors of all-cause in-hospital mortality. Furthermore, a level of 2.2 to ≤2.4 of serum magnesium showed a higher risk of in-hospital mortality compared to a level of more than 2.4 mg/dL [12].

One study revealed that serum magnesium level was lower among AMI patients with complications compared to those without complications [6]. In our study, patients with certain complications significantly experienced low serum levels, and those were patients who experienced atrial fibrillation, angina, and cardiogenic shock. On the other hand, other complications, including ventricular tachycardia, ventricular fibrillation, thrombotic events, and sustained premature ventricular beats, did not show significant variation between patients with low and normal serum magnesium levels.

Limitations, strengths, and recommendations

The limitations of this study include conducting the study at one center, and we did not use a multivariate analysis for the assessment of low magnesium levels as a risk factor for adverse outcomes. The strength of the study included a simple study with clear findings, and it is the first Saudi study conducted on this subject as far as we know. Further studies are recommended to be conducted on this subject.

## Conclusions

Most acute myocardial infarction patients experience a low level of serum magnesium on the first day of admission at the hospital. The low level of serum magnesium is associated with developing other complications, including atrial fibrillation, angina, and cardiogenic shock. However, no patient was reported to have a complex arrhythmia.

The future perspective of this study is that the study highlighted the importance of assessing levels of serum magnesium among acute myocardial infarction patients. This may mean that the level of serum magnesium can be used as a predictor for poor or good acute myocardial infarction outcomes. Additionally, this may suggest using magnesium for the treatment of acute myocardial infarction. However, this requires further investigation.
